# Clinical and immuno-proteomic approach on *Lantana camara* pollen allergy—a major health hazard

This article has been retracted.

**DOI:** 10.1186/s13223-016-0135-z

**Published:** 2016-07-28

**Authors:** Kavita Ghosal, Bodhisattwa Saha, Swati Gupta Bhattacharya

**Affiliations:** Division of Plant Biology, Bose Institute, Main Campus, 93/1, A.P.C. Road, Kolkata, West Bengal 700009 India

**Keywords:** Aero-allergen, *Lantana camara*, Statistical analysis, 2D Gel electrophoresis, Immunoblot, MALDI-TOF/TOF

## Abstract

**Background:**

The incidence of allergic diseases is increasing gradually and is a global burden affecting the socio-economic quality of life. Identification of allergens is the first step towards paving the way for therapeutic interventions against atopic diseases. Our previous investigation figured out that total pollen load correlated significantly with the rise of respiratory allergy in a subtropical city in India. The most dominant pollen responsible for IgE sensitivity in most patients emerged to be from *Lantana camara* (LC) an obnoxious weed growing in and around suburban areas of West Bengal. In this study, we identified allergenic components from this shrub using an immunoproteomic approach.

**Methods:**

Determination of dominant pollen species was done using aerobiological sampling during two consecutive years and correlated with hospitalization and skin prick test. Serum was collected from LC positive patients and checked for in vitro allergenicity using ELISA and Histamine assay. Total proteome was profiled in SDS–PAGE, 2D PAGE and immunoblotted to detect IgE binding proteins which were further identified using mass spectrometry.

**Results:**

*Lantana camara* pollen emerged as a significant contributor from the correlation study with hospital admission of the respiratory allergy sufferers and its extract demonstrated an elevated IgE response in ELISA and histamine release assay tests. Five IgE reactive bands/zones were observed in 1D blot which resolved to 12 allergo-reactive spots in the 2D blot. Mass spectrometric analysis identified nine spots that grouped into four diverse proteins. Pathogenesis-related Thaumatin-like protein was found to be one of the major allergens in *Lantana camara.*

**Conclusions:**

This is to our knowledge the first attempt to identify allergens from *Lantana camara* using a proteomic approach. The allergens identified thereof can be used to prepare hypoallergenic vaccine candidates and design immunotherapy trials against LC pollen and other aeroallergen carriers which are cross-reactive and harbor similar proteins.

**Electronic supplementary material:**

The online version of this article (doi:10.1186/s13223-016-0135-z) contains supplementary material, which is available to authorized users.

## Background

Allergic diseases are amongst the most chronic disorders worldwide [1]. Presently, 300 million people are reported to suffer from one or more allergic diseases, affecting the socio-economic quality of life [2]. About 20–30 % of the total population suffers from various types of allergic diseases in India [3] and is ascending in terms of preponderance as well as severity. Pollen grains are one of the major aeroallergen carriers and are well known to trigger respiratory allergies and asthma in predisposed individuals [4, 5].

Our previous 2 years aero-palynological study in Konnagar, a subtropical suburban city of India for their prevalence in the atmosphere revealed noteworthy interrelationship between total airborne pollen load and type-1 hypersensitivity related symptoms [6]. Phenotypic manifestations were documented from the chest and respiratory unit of a local hospital accompanied by a regional health survey. The study reported the presence of different pollen species, mostly members from Arecaceae, Poaceae, and their seasonal distribution. Amongst these, *Lantana camara* (LC) was found to contribute a significant proportion of aero palynological load (Additional file 1) and atopicity as revealed by skin prick tests (SPT). This prompted us to investigate its allergenic potency and identify the IgE sensitive components in more detail.

*Lantana camara* (Family: Verbenaceae) commonly known as red sage, the most widespread species of the genus is a noxious weed and reported as one of the top ten worst weeds in the world [7]. A native of South and Central America, it is tolerant to a wide range of ecological niches and is listed amongst the top invaders in India. However, though, it has a few medicinal uses. Extracts of LC leaves has been used as folk medicine for antiseptic, antimalarial, antitumoural, antimicrobial activity [8, 9] and insecticidal properties [10]. Allergenicity to LC pollen is relatively new. A previous study reported LC pollen is responsible for IgE sensitivity amongst approximately 8 % out of a cohort of 1500 patients in Kolkata, a megacity of India. Further, four IgE reactive bands have been described along with its chemical composition in terms of lipid, carbohydrate and protein content as well as cross-reactivity amongst other Verbenaceae pollen taxa [11]. LC pollen was also found to cause allergenicity in 5 % of atopic patients in a city of North India [12].

The last decade has seen unprecedented developments in allergen identification from various pollen grains using different techniques. Amongst these, proteomics platform has helped to identify allergens rapidly compared to other methods such as cDNA expression library screening, amino acid micro-sequencing to name a few. Allergens from *Lolium perenne* [13], Coconut [14], Sunflower [15] pollen grains have been successfully identified by immunoproteomic approach. 2D gel electrophoresis resolves protein complexes into individual proteins much precisely compared to normal SDS–PAGE as well as distinguish isoforms assisting in accurately identifying the protein of interest. To determine the allergens from LC pollen more definitively we have employed a similar immunoproteomic study. Total pollen extract was profiled in a 2D gel and immunoblotted with pooled patient sera. Immunoreactive spots were identified and subjected to mass spectrometry for allergen identification. LC being unsequenced, we have employed a proteomic workflow combining conventional database dependant search as well as de novo sequencing to decipher the identity of the IgE sensitive spots. Further individual patient reactivity has been demonstrated through histamine release and specific IgE (sIgE) ELISA tests. To the best of our knowledge, this is the first comprehensive report to identify allergens from LC.

## Methods

### Survey in hospital

Clinical data of an overall 1082 patients suffering from allergic rhinitis, lower and upper respiratory tract infections and bronchial asthma along with their rate of hospitalization were documented from Kamala Ray Hospital near the research site.

### Determination of patients-pollen correlation

To verify whether the LC pollen is having an impact on patients’ hospitalization, statistical correlation has been performed for LC pollen with patients’ hospitalization data. Spearman’s non-parametric correlations have been followed at 95 % confidence level employing the statistical package for the social sciences (SPSS) 20.0 software. Multiple linear regression analysis further confirmed the correlation.

### Collection of pollen sample

Fresh pollen grains were collected from immature buds and mature flowers of LC growing in and around the study area during their peak blooming period. They were air dried, mildly crushed and passed successively through sieves of decreasing pore size until 90–95 % purity pollen was obtained.

### Preparation of LC pollen extracts for SPT

One hundred and fifty milligram pollen grains were defatted with diethyl ether to remove pigment on the outer pollen surface and crushed to powder in liquid nitrogen. Ground pollen was incubated in 2 ml of 0.1 M Phosphate Buffer (pH 7.2) under constant shaking at 4 °C overnight. Thereafter, the slurry was centrifuged at 22,000×*g* for 20 min at 4 °C to collect the supernatant. Subsequently, the supernatant was passed through Main Flow Bacterial/Viral Filter (Telefax, USA) and applied for SPT. Protein concentration was estimated with Bradford reagent (Bio-Rad, USA).

### Patient selection and sera collection

Adult patients (>18 years) suffering from allergic rhinitis, bronchial asthma, rhinoconjunctivitis and substantial history of seasonal pollen allergy were included in the study. Individuals undergoing immunotherapy trials or under antihistaminic medication, immune-compromised subjects, breastfeeding women and smokers were excluded. Skin prick tests were done with antigenic extract using a sterile lancet and graded as described previously [16]. Histamine diphosphate (1 mg/ml) and Phosphate buffer (0.01 M, pH 7.2) were used as positive and negative controls respectively. 96 out of 150 patient cohorts showed a positive cutaneous response to LC pollen extract. Out of them, 15 individuals with high SPT grades (>+3) and total IgE agreed to provide blood for further immunobiochemical assays on a written consent. Sera from six nonatopic individuals were used as negative control. 5 ml of blood was collected from each patient; serum was separated and stored at −80 °C until use.

### Total protein extraction from LC pollen

One gram of defatted crushed sample was mixed with acetone containing 10 % trichloroacetic acid (w/v) and 1 % dithiothreitol (DTT) (w/v), under constant shaking at 4 °C overnight. Thereafter, it was centrifuged at 22,000×*g* for 20 min at 4 °C. The pellet was cleaned twofold by suspending in acetone containing 1 % DTT, 0.01 % protease inhibitor cocktail (Sigma, St Louis); kept at −20 °C for 1 h and centrifuged. The supernatant was discarded, and the pellet was vacuum dried. For 1D gel electrophoresis, the pellet was dissolved in 0.1 M Phosphate Buffer (pH 7.2). For 2D electrophoresis, isoelectric focusing buffer (IEF) was added in sufficient amount to submerge the pellet and incubated overnight at −20 °C. The supernatant was collected by centrifuging it at 22,000×*g* for 20 min at 4 °C. The extract was mixed with Protease inhibitor cocktail (Sigma, St Louis) at 0.01 % of the total extract volume accordingly [17]. Quantitative estimation of protein was done as mentioned before.

### 1D sodium dodecyl sulfate–polyacrylamide gel electrophoresis (SDS–PAGE)

Ninety microgram of total protein was resolved on 12 % SDS–PAGE under denaturing condition using a vertical gel electrophoresis apparatus (GE Life Sciences, USA) along with a standard protein molecular weight (MW) marker (GeNei, India). The protein bands were observed by Coomassie Brilliant Blue-R250 (CBB-R250) staining.

### 2D Gel electrophoresis

Protein suspended in IEF buffer was cleaned using Focus Perfect^TM^ 2D Cleanup Kit (G-Biosciences, USA) to remove impurities such as salts and detergents. 400 μg sample was reconstituted freshly in 125 μl IEF buffer with 1 % immobilized pH gradient (IPG) pH 4–7 linear buffer (v/v) (GE Healthcare, Sweden), 25 mM DTT and 0.002 % Bromophenol blue. Rehydration loading was done on a 7 cm immobiline dry strip (Amersham Biosciences, USA) in a reswelling tray overnight at room temperature. Isoelectric focusing was achieved using Ettan IPGphor 3 (GE Healthcare). Thereafter the strip was equilibrated in equilibration buffer-I (6 M Urea, 75 mM Tris–HCl pH 8.8, 30 % glycerol, 2 % SDS and 1 % w/v DTT) for 15 min followed by equilibration buffer-II (same as equilibration buffer-I with 2.5 % w/v iodoacetamide instead of DTT).Finally, the strip was laid on a 12 % SDS–PAGE gel and stained in CBB R250.

### IgE specific 1D and 2D western blot

IgE specific western blotting was done according to the protocol described previously [18]. Total protein profile in 12 % SDS–PAGE was transferred to a polyvinyl difluoride membrane (PVDF) (GE Life Sciences, USA) by semi-dry transfer method through a constant current of 1.2 mA/cm^2^ for 1 h. Transfer of bands/spots to the membrane was ensured by staining in Ponceau S. Blocking was done with Tris Buffered Saline +0.05 % tween-20 containing 3 % bovine serum albumin (TBST-BSA) for 3 h at 4 °C. Primary antibody incubation was done using fifteen individual sensitive patients’ sera diluted in 1:10 ratio in blocking solution at 4 °C. After washing thrice with TBST, incubation was done with monoclonal anti-human IgE alkaline phosphatase tagged produced in a mouse (Sigma) in 1:1000 dilutions in blocking solution as a secondary antibody. Reactive bands were detected by addition of NBT-BCIP (nitro blue tetrazolium chloride-5-bromo-4-chloro-3-indolyl-phosphate) (Sigma), and the reaction was stopped with 0.5 M ethylenediaminetetraacetic acid (EDTA).

For 2D blotting, the spots from the 2D gel were transferred to LFT-PVDF membrane in a similar way according to 1D blot. After transfer, the membrane was incubated with pooled sera of LC positive patients as done previously [19].

Gels for 2D blotting and staining were run parallel with same protein loads and experimental parameters to ensure IgE reactive spots in blot exist in the same coordinates of the stained gel. Further, the spots in gel, membrane stained with Ponceau S and immunoblot were compared visually as well as in Image Master 2D (GE Lifesciences) to reduce false positives. Molecular weight and pI was determined in Quantity One Software (Bio-Rad).

### Sample preparation for mass spectrometry

Sample preparation was done following a protocol described by Shevchenko et al. [20] with minor modifications. IgE reactive spots corresponding to 2D blot were excised with sterile scalpels and destained in 50 mM ammonium bicarbonate (ABC) (pH 8.0) containing 50 % ethanol followed by reduction and alkylation with 10 mM DTT (Sigma) and 55 mM iodoacetamide (Sigma) respectively. After that gel pieces were rehydrated and dehydrated in 50 mM ABC and 100 % acetonitrile (ACN) respectively. In-gel digestion was carried out in 12.5 ng/μl of trypsin (Trypsin Gold, Promega, USA) at 37 °C for 16 h. After removing trypsin, peptides were extracted from gel pieces by vigorous vortexing in extraction buffer composed of 30 % ACN and 1 % Trifluoroacetic acid. The extracted peptides were dried in a speed vac (Savant, USA). About 1.5 μl peptide digests were mixed with equal volume of 0.5 mg/ml α-cyano-4-hydroxycinnamic acid (HCCA) matrix solution (Bruker Daltonics, Germany) and was dotted onto MTP 384 ground steel target plate (Bruker) and air dried.

### Mass spectrometric (MS) analysis

Mass spectra were acquired with Autoflex II matrix-assisted laser desorption/ionization—time of flight (MALDI TOF/TOF) (Bruker Daltonics) and peptide monoisotopic signals were analyzed in Flex Analysis software (version 3.0, Bruker Daltonics) through manual data acquisition. MS/MS was done by manually selecting high-intensity precursor ions and fragmenting in LIFT mode with 4000–8000 laser shots. The parent and daughter ions were analyzed using SNAP algorithm of the Flex Analysis software (version 3.0, Bruker Daltonics). Spectral baseline subtraction, smoothing, and centroiding were performed by Flex Analysis Software v3.0. The processed peaks were conveyed through MS BioTools™ (version 3.0) as inputs to the MASCOT (http://www.matrixscience.com) search engine, version 2.2 for protein identification. The following parameters were set for MASCOT-search, Database: National Center for Biotechnology Information Nonredundant (NCBInr) (1,438,958 sequences, Dec 2015); Taxonomy: Viridiplantae; Proteolytic enzyme: trypsin; mass tolerance of precursor ions and fragments were set to 1.2 and 0.5 Da respectively; global modification: carbamidomethylation of cysteine; variable modification: oxidation of methionine; maximum missed cleavage of 1. Protein identifications were considered reliable once the identification was considered confident (p < 0.5). Common contaminants such as keratin, trypsin autolysis, and matrix peaks were eliminated by an internal calibration in Flex analysis software.

### Manual de novo sequencing

The spots that could not be identified by database dependant search were sequenced manually from the spectra using preset rules as described previously [21, 22]. Sequencing was done employing difference of mass approach using the annotation tool in Flex analysis (Bruker) primarily by locating high intensity “y” ions. Sequence proposals generated from the de novo sequencing of each MS/MS spectra was used for similarity searches using the MS-BLAST algorithm (http://www.genetics.bwh.harvard.edu/msblast/) through online submissions. Searches were performed using the settings, Program: Blast 2p; non-redundant database (nr 95 2014_01); matrix as Point Accepted Mutation (PAM 30); “Expect” as 100.

### Indirect enzyme-linked immuno-sorbent assay (ELISA)

50 µl/well of LC pollen extract (100 ng/µl) were coated on ELISA plate (Nunc, Denmark) and incubated overnight at 4 °C. After washing thrice with Phosphate Buffered Saline containing 0.05 % Tween 20 (PBST) wells were blocked with 1 % Bovine serum albumin (BSA) diluted in PBST at 4 °C as previously described [23]. Incubation in primary antibody was done at 4 °C using sera diluted 1:10 from patients or non-atopic controls. Monoclonal anti-Human IgE alkaline phosphatase tagged, produced in a mouse (Sigma) was used as secondary antibody diluted 1:1000 and incubated at 37 °C for 3 h. Wells were then incubated in para-nitrophenyl phosphatase (pNPP) for 30 min at 37 °C in dark and OD values were recorded in ELISA reader (Multiskan, Thermo) at 405 nm. Experiments were done in triplicates and mean values represented.

### Stripped basophil histamine-release assay

Histamine-release assay was performed as previously described [24]. In Brief, peripheral blood was collected from nonatopic controls, and peripheral blood mononuclear cells were separated by Ficoll Paque (GE Lifesciences). Stripping of bound IgE from basophils was done by incubation in lactic acid buffer (13.4 mM lactate, 140 mM NaCl and 5 mM KCl at pH 3.5) for 3 min followed by washing in 4-(2-hydroxyethyl)-1-piperazine ethane sulfonic acid (HEPES) buffer (pH 7.5) and resensitized in sensitization mixture (150 μL, 4 mM EDTA sera from 10 allergic patients) at 37 °C for 90 min. Thereafter, cells were allowed to recover in 2 ml of HEPES buffer containing 1 mM CaCl_2_ (30 min, 37 °C) and then stimulated with 1 μg of crude allergen diluted in 100 µl of HEPES buffer containing 1 mM CaCl_2_ for 1 h at 37 °C. The reaction was then stopped by the addition of ice-cold 0.9 % NaCl (w/v) and cells pelleted at 12,000 g for 3 min. The supernatant was mixed with 200 µl of perchloric acid and used for histamine estimation. Cells sensitized with two non-allergic sera were taken as controls. BSA was used as a negative control. The total histamine content was determined by lysing cells after repeated freeze–thaw cycles. Spontaneous histamine release was measured in the supernatant of unstimulated cells without allergen challenge [14]. Histamine content was evaluated through competitive ELISA according to the manufacturer’s instructions using Enzyme immunoassay (EIA)–Histamine assay kit (Immunotech, France). Linear regression analysis with total histamine release assay and IgE specific ELISA of LC has been performed following Spearman’s correlation analysis.

### Statistical analysis

A heat map was created using R statistical computing package (version3.1.1) by initially converting IgE reactive bands into a binary matrix as presence or absence in different patients [25]. Both row and column clustering was done according to the Euclidean distance to arrange patients and allergenic bands into groups for ease of analysis. All other statistical analysis was done in Prism 6 software (Graphpad).

## Results

### Determination of most prevalent respiratory ailment from hospital survey

It has been found from patients’ records that allergic rhinitis scored highest with 55 % followed by asthma with 26 % sufferers during the survey period. Additionally upper and lower respiratory tract infections were also prevalent (Fig. 1a). The data also revealed that female and passive smokers were more in number than male and active smokers in hospitalization (Fig. 1b, d). Patients less than 40 years were most susceptible followed by the patients less than 60 and 15 years respectively (Fig. 1c).

**Fig. 1:** Comparative accounts for the interpretation of the hospital data and pollen counts. **a** Doughnut chart of various types of respiratory diseases in percentages (%) according to patients’ admission. **b** Male–female comparison from hospital survey. **c** Age group comparison from hospital survey. **d** Active–passive smoking comparison from hospital survey. **e** Comparative graph showing the blooming period of *Lantana camara* and patients hospitalization during 2010–2011 and 2011–2012

### Correlation study between LC pollen counts and patients’ admission

The LC pollen counts showed a significant positive correlation with the total patients’ admission data in the two consecutive years of 2010–2011 and 2011–2012. Their correlation values were 0.993 and 0.986 (p <0.01 level) in the 2 years accordingly. Linear regression analysis confirmed this correlation. The results were statistically significant with an adjusted r^2^ value of 0.802 (2010–2011) and 0.816 (2011–2012), which accounted for approximately 80.2 and 81.6 % of the variance in patients’ hospitalization in the 2 years (Additional file 1). Besides, LC showed a better correlation in terms of blooming period and patients’ admission (Fig. 1e).

### SDS-PAGE and immunoblot

LC pollen extract separated in 1D PAGE revealed approximately 29 bands within the MW of 14.3–97 kDa. Upon immunoblotting with each of 15 patient specific sera, five distinct IgE reactive bands at 30, 38, 45, 51, and 67 kDa was noticed. In addition, an IgE sensitive region was observed between 25 and 27 kDa which could not be distinctly identified as individual bands due to their close spacing (Fig. 2a). No allergens were detected in the control patients and are shown alongside.

**Fig. 2:** 1D Immunoblot displaying sIgE reactive bands and their frequency in Cluster analysis. **a** 1D electrophoresis and IgE specific Immunolbot with LC sensitive patient sera. *Lane M* molecular marker; *Lane C* Crude extract of LC pollen in 12 % SDS–PAGE, *Lane 1–15* IgE specific Immunoblots with 15 patients’ sera, *C1–C6* negative control with sera of non atopic patients. **b** Graphical representation of cluster analysis showing the frequency of seven IgE reactive bands. *A* Minor allergens, *B* Major allergens; ~25–27 and ~30 kDa were present in highest frequency and therefore considered the major allergen; *I* Most sensitive, *II* intermediate sensitive patients, *III* Most sensitive towards major allergens

### Identification of major and minor allergenic bands by cluster analysis

Figure 2b illustrates a heat map generated by hierarchical cluster analysis based on the presence and absence of IgE reactive bands in fifteen 1D immunoblots representing individual patient sensitization profile. Column clustering sorted the bands into two groups: A and B. Group A comprising bands of the 25–27 kDa region, ~30, ~45 and the ~51–52 kDa zone were found to be seroreactive in more than 70 % of the patients. Amongst them the 25–27 kDa region and 30 kDa IgE reactive band were IgE reactive in all patients under study and are considered to be major allergens. Group B representing an allergen cluster composed of 36 and 67 kDa protein bands were less reactive compared to group A and recognized as minor allergens.

Row clustering classified all the 15 patients into three groups I, II and III. Group I which include 40 % of patients, was highly sensitive to almost all the LC allergens. Group II includes 33 % of patients displaying strong IgE reactivity to the major allergens and less reactivity with other allergens. Group III patients showed reactivity only with the major allergens but no reactivity towards minor allergens.

### 2D gel electrophoresis and 2D immunoblot

Total pollen proteome was resolved in narrow range 2D gel which helped to separate closely spaced bands into more than 120 individual protein spots within 4–7 pH range and MW of 14–97 kDa regions (Fig. 3a). Most of the immunoreactive proteins were ranging from 19 to 70 kDa and were in between acidic to neutral pI. Few spots such as 3, 7 and 8 were well separated from each other while others were present in a string of spots having almost same molecular weight but different pI in three different molecular weight regions, approximately at 45, 51 and 67 kDa respectively (Fig. 3b). 2D immunoblots with individual patient sera could not be performed due the scarce availability of sera. None of the proteins displayed reactivity with pooled control serum (Fig. 3c).

**Fig. 3:** Identification IgE reactive proteins from the two dimensional map of *Lantana camara.* **a** 2D gel profile of the total protein extracted from LC and marked with *arrows* of IgE reactive. spots corresponding to immunoblot analysis; M: molecular marker, **b** 2D-IgE specific immunoblots revealed IgE reactive spots in 7 cm gel. **c** 2D immunoblot with healthy patient sera as negative control

### Identification of allergens by mass spectrometry

9 out of 12 IgE reactive protein spots could be identified by MALDI-TOF/TOF based on homology with other plant taxa (Table 1) Identifications were considered confident when at least two unique peptides scored above the threshold level (p < 0.05). Through MASCOT search against NCBI database spot 1 and 2 showed homology with Actin; spot 4, 5 and 6 with Adenosine triphosphate (ATP) synthase beta subunit respectively. In the case of spot 3, 7 and 8 only one unique peptide from each spot showed homology with Thaumatin-like protein (TLP) (Fig. 4c). One peptide from each of spot 3 and 8 was identified as hypothetical proteins on conventional MASCOT search. These peptides showed similarity with TLP from *Sesamum indicum* upon NCBI BLASTp using default settings. For the remaining peptides, whose MASCOT score was below significance, were de novo sequenced manually and interpreted in MS-BLAST through homology-based search without taxonomic restriction. This led to few more peptide annotations in spot 7 and 9. De novo sequencing for two peptides of m/z 2169.09 and 1683.775 Da of spot 7 derived the sequence to be “RLDSGQSWQVNVAARVRAR” and “NQQCPNEI/LRN” (Fig. 4a, b). Homology-based search with MS BLAST showed considerable similarity with TLP (Fig. 4c, d). Similarly, another unique peptide of m/z1360.786 from spot 9 identified the sequence to be “HNEFELSDTLR” showing homology to Glutamate decarboxylase (Fig. 5). Due to the low intensity of spot no: 10, 11, 12 of 75 kDa proteins, no significant results could be derived from mass spectrometry. The result of MASCOT search for all the peptides is described in the Additional file 2.

**Table 1:** Identification of allergens from *Lantana camara* pollen grains using MALDI TOF/TOF

SN	Identified protein^d^	Organism	Accession no.	Identified peptides^b^	E value^a^	Expt. MW/pI	Theor. MW/pI	Score	UP^b^	Seq. cov. (%)
1.	Actin	*Glycine max*	CAA23728.1	KIWHHTFYNELRV	0.0019	45.6/5.8	41.56/5.23	64	2	3.45
		*Maurandya* *barclaiana*	AAL89713.1	KSFELPDGQVITIGNERF	6.2e−05		19.996/5.02	78		9.94
2.	Actin	Glycine max	CAA23728.1	KIWHHTFYNELRV	0.00017	45.6/5.8	41.56/5.23	69	3	3.45
		*Chlorella vulgaris*	AAB07499.1	KSYELPDGQVITIGNERF	1.3e−05		23.18/4.89	83		8.78
		*Phaseolus vulgaris*	AGV54465.1	RTTGIVLDSGNGVSHTVPIYEGYALPHAILRL	0.0037		41.66/5.39	50		8.48
3.	TLP; Ole e 13	*Olea Europea*	E3SU11.1	RCPDAYSYPQDDPTSLFTCPAGTNYRV	1.3	19.4**/**4.2	24.7/5.1	31	2	11.94
	HP	*Erythranthe guttata*	EYU38379.1	RCTAPINEQCPNELRA	0.075		24.9/5.3	42		6.95
4.	F1ATPase	*Pisum sativum*	BAA20135.1	KTEHFLPIHRE	0.014	51.8/5.5	60.1/6.6	52	3	1.96
	ATP Synthase subunit beta	*Nicotiana plumbaginifolia*	CAA26620	RFTQANSEVSALLGRI	0.027		59.8/5.9	48		2.85
		*Tricum aestivum*	CAA52636.1	RLVLEVAQHLGENVVRT	0.013		59.24/5.5	50		3.07
5.	ATP Synthase beta subunit	*Tricum aestivum*	CAA52636.1	RLVLEVAQHLGENVVRT	0.046	51.8/5.6	59.2/5.56	44	2	3.07
		*Nicotiana plumbaginifolia*	CAA26620.1	RDAEGQDVLLFIDNIFRF	0.0077		59.85/5.95	56		3.21
6.	*ATP Synthase* beta subunit	*Triticum aestivum*	CAA52636.1	RLVLEVAQHLGENVVRT	0.43	51.84/	59.24/5.56	38	2	3.07
		*Nicotiana plumbaginifolia*	CAA26620.1	RDAEGQDVLLFIDNIFRF	0.29	5.7	59.85/5.95	40		3.21
7.	TLP; Ole e 13	*Olea Europea*	E3SU11.1	RCPDAYSYPQDDPTSLFTCPAGTNYRV	5.1e−13	21.85/6.5	24.72/5.10	150	3	11.94
	Predicted TLP	*Solanum Lycopersicum*	XP_004252644.1	RLDSGQSWQVNVAARVRAR	NA^c^		45.53/4.95			4.55
	PRP	*Solanum tuberosum*	XP_006364119.1	NQQCPNELRN	NA^c^		25.00/5.31			4.4
8.	TLP; Ole e 13	(*Olea Europea*)	E3SU11.1	RCPDAYSYPQDDPT SLFTCPAGTNYRV	5.9e−06	19.28/6.159	24.72/5.10	79	2	11.94
	HP	*Erythranthe guttata*	EYU38385.1	RCTAPINEQCPNELRA	0.018		81.11/8.03	48		2.2
9.	Predicted GAD 1- like	*Glycine max*	XP_003544967.1	KVLHELDLLPARV	0.94		52.685/5.831	34	2	2.58
	GAD	*Nicotiana tabacum*)	AAM48129.1	HNEFELSDTLR	NA^c^					2.21

^a^Probability score at the <0.05 level

^b^UP, unique peptides have been identified by MASCOT search against NCBI database

^c^Manual de novo sequencing has been performed for the respective peptide sequence

^d^Identified proteins: actin, TLP, thaumatin like protein; HP, hypothetical protein MIMGU_ngvla013131 mg; PRP, pathogenesis related protein, GAD, glutamic acid decarboxylase

**Fig. 4:** De novo sequencing from the spot no: 7. **a**, **b** De novo sequencing of peptide m/z: 1683.77 and 2169.09 Da from the spot no: 7; the derived sequences are mentioned on the *top* of the spectra.. **c** MASCOT result of peptide 2895.34 Da showing similarity with allergen Ole e 13 from Olive also described as Thaumatin like protein (TLP). **d** Result of MS-BLAST with the two derived peptides 1683.77 and 2169.09 Da demonstrating significant homology with (TLP) from *Solanum lycopersicon*. C* carbamidomethylated cysteine

**Fig. 5:** De novo sequencing from the spot no: 9. **a** De novo sequencing of Peptide m/z: 1360.786 Da from the spot no: 9 The derived sequence is mentioned on the *top* of the spectra. **b** Result of MS-BLAST with the peptide 1360.786 Da demonstrating significant homology with Glutamate decarboxylase from *Nicotiana tabacum*

### Indirect ELISA and histamine release assay

LC sensitive patient sera with +2/+3/+4 skin reactivity showed elevated specific IgE compared to nonatopic controls (Table 2). Group 1 patients showed sixfold and other patients showed fourfold higher IgE reactivity compared to controls respectively (Fig. 6a). Histamine release upon challenging basophils with crude LC extract was significantly elevated (p < 0.05) in the range of 49–70 % of the total histamine. In the case of control sera, histamine release varied between 4 and 9 %. BSA as a negative control also showed low histamine release (Fig. 6b). There was no significant difference between group II and III patients in both ELISA and histamine release. Patients with high specific IgE also had higher SPT values. A positive correlation with a high linear regression coefficient (r^2^ value: 0.86) was observed between histamine release and specific IgE (Fig. 6c).

**Table 2:** Result of SPT, histamine release assay and IgE specific ELISA

Patient no	Age/sex	Symptoms^a^/clinical history	Aeroallergen^b^ sensitization/SPT grade^c^ for *Lantana camara*	Histamine release in cell (concentration nM)	Specific IgE-ELISA for *L. camara* (OD value)^d^
1	18/F	AR, SOB	CN, LC/(+3)	1912.973	2.8
2	30/M	AR	AC, LC/(+3)	1001.521	2.76
3	25/M	AR + BA, SOB	GP, TG, LC/(+3)	768.489	2.66
4	31/F	AR + BA	AF, AI, LC//(+4)	1500.347	3.1
5	27/F	AR, SOB	AC, CN, LC/(+4)	817.62	3.32
6	16/F	AR + BA	HD, AF, LC/(+4)	623.983	2.92
7	37/M	AR	CP, TG, PS, LC/(+3)	737.714	3.06
8	34/F	AR, SOB	AI, CP, LC/(+2)	1999.624	2.43
9	41/M	AR + BA, SOB	GP, PS, LC/(+3)	915.651	2.95
10	42/F	AR + BA, SOB	PS, LC,/(+3)	1280.903	2.67
11	34/F	AR + BA	CN, LC/(+4)	676.54	3.4
12	30/M	AR	CN, PS, LC/(+3)	1622.213	2.79
13	35/M	AR, SOB	GP, LC/(+2)	814.312	2.37
14	41/M	AR	AC, CN, LC/(+3)	1315.149	2.76
15	22/F	AR	GP, LC/(+3)	1722.743	3.00
Control					
1	25/F	AR + BA	AI, AF/(+3)	31.619	0.847
2	15/F	AR	CP, CN/(+2)	10.237	0.912
3	23/M	AR + BA	HD, AI/(+3)	80.143	1.105
4	30/F	AR	CP, PS/(+3)	62.358	1.131
5	28/M	AR + BA	CN, HD/(+2)	19.186	0.984

^a^Symptoms: *AR* allergic rhinitis, *BA* bronchial asthma

^b^Aeroallergens: AC, *Areca catechu*; AF, *Aspergillus flavus*; AI, *Azadirachta indica*; CN, *Cocos nucifer*a; CP, *Carica papaya*; GP, grass pollen; HD, house dust; LC, *Lantana camara*; PS, *Phoenix sylvestris*

^c^Reactions in SPT: +no wheal and erythema of 20 mm in diameter; ++wheal and erythema of 20 mm in diameter; +++wheal and erythema >30 mm; no wheal and no erythema; control group had P/N value <1.5

^d^P/N: ratio of optical density of patient serum with respect to control

**Fig. 6:** Allergenic Potency of *Lantana* pollen extract and its major allergen. **a** Specific IgE ELISA. *Dot plot* showing the distribution of group specific IgE titers among 15 patients due to crude allergen extract along with IgE titers. **b** Stripped basophil histamine release assay. Grouped distribution showing histamine release due to crude allergen; control and BSA: Negative control. Statistical analysis: two-way ANOVA employing Bonferroni multiple comparisons test. *Represents significance at p < 0.05. Specific IgE titers were significant in *pairs* and across *columns*. Patients of Group 1 (1, 8, 15, 12, 10, 14) showed elevated histamine release compared to others. **c** Linear regression model following Spearman’s correlation of total histamine release in cell and sIgE-ELISA of *Lantana camara*. Correlation coefficient (r) value: 0.8007; p value: 0.003 where correlation is significant <0.005 level

## Discussion

Allergic disorders are gradually increasing in India due to urbanization. *Lantana camara* is an obnoxious weed and has been found widely growing in suburban areas of eastern India. This species has been found to colonize the area in which it grows by replacing the native species uncontrollably [7, 26] leading to a release of a substantial amount of pollen grains in the atmosphere which reaches maximum during the period between November to May causing allergic sensitization in predisposed individuals. The present investigation is focused on allergenicity assessment of *Lantana camara* pollen, the most predominant pollen species contributing to atopic diseases in susceptible patients in Konnagar, suburban city of eastern India through clinical survey and ascertaining its allergenic components by an immunoproteomic approach. Currently, atopic diseases are treated through antihistamines, steroidal drugs which have their inherent side effects. The only remedy able to cure allergic diseases and to confer long-lasting protection remains allergen-specific immunotherapy (SIT) using hypoallergenic candidates. Identification of relevant allergens from various sources is primarily required for the development of such therapeutic interventions.

A shortcoming in 1D blot is that a band does not necessarily mean single protein as it may contain isoforms of a single protein or many proteins having different isoelectric points. 2D gel resolves the proteome in terms of MW and pI helping to distinguish individual proteins and facilitating their identification by mass spectrometry. Due to limited availability of sera, 2D blots with individual sera could not be performed. The six immunoreactive bands resolved into 12 spots in the 2D gel (pI 4–7). LC pollen proteome was initially profiled in a 3–10 pI gel but it was observed that most of the proteins were concentrated in the 4–7 region as well as the IgE-reactive spots (Data not shown). So, further experiments were done in the 4–7 pI gels. Similar 2D immunoblot with pooled sera was done to identify allergens from *Plantago lanceolata* and detect the presence of isoforms or protein complexes in an IgE binding hotspot observed in 1D blot [27].

IgE reactive bands between 25 and 27 kDa resolved into two spots with pI 4 and 6. The 30 kDa band had a single spot in that region whereas the other three bands of 45, 51 and 67 kDa had more than one spot. All the IgE-reactive bands correlated well with corresponding reactive spots on 2D blot except for 36 kDa band. This protein was found to be positive in only three patients and did not appear in 2D blot, which can be assumed by the fact of restricted protein loading in the 2D gel and limited IgE antibodies of the corresponding patients in the pooled sera. Each band in 1D blot corresponded to a single kind of protein, some of which were in isoforms. Even though 1D blot could not identify the individual allergens the heatmap generated thereof gives a rough blueprint of each individual patient reactivity profiles.

Patients in group I was found to be highly allergenic to LC extract in terms of high specific IgE values and histamine release. These patients also showed IgE reactivity to most of the allergens detected in this pollen grain. Other patients who recognized fewer IgE bands had moderate IgE sensitivity and histamine release. The absence of significant difference in IgE titer and histamine between group II and III suggests their equal allergenic response to LC pollen allergy. A positive correlation was seen between immunoblots, specific IgE and histamine inferring relatedness in the in vitro allergenicity assays. This also suggests that the IgE binding is probably dominated by linear epitopes in LC pollen grains.

One of the major bottlenecks of proteomics is that it depends entirely on the presence of complete protein databases. A change in a DNA base ultimately may change an amino acid which has a deep impact on the mass of peptide causing the scores to decrease lower than significance. Hence, it becomes difficult to identify the proteins from unsequenced genomes. In identifying the allergens from LC pollen, a database search was used as the first screening step to identify proteins which are highly homologous or identical to those in the database. Peptides which were vaguely or unidentified in MASCOT search were de novo sequenced directly from spectra and the sequence proposals generated thereof were searched for similar or homologous peptides. Homology search relies on similarity, not identity which can be accomplished by allowing multiple mismatches in a sequence stretch [28]. The combination of database dependant and homology-based search helped to increase the query coverage and a number of unique peptides thus reinforcing the results. For example, in spot 7 peptide 2169 and 1683.77 Da did not give reliable results in MASCOT search. De novo sequencing of these peptides generated a few peptide proposals of which N’ RLDSGQSWQVNVAARVRAR’C and N’… NQQCPNELR C’ showed similarity with TLP from *Solanumlycopersicum* from MS BLAST search. In the output result of 2169 Da peptide from MS BLAST, several mismatches between the query protein and sequenced peptide could be noticed at the 7th, 9th and 10th position changing threonine to serine, asparagine to glutamine, isoleucine to valine. It is evident that such changes occur due to single nucleotide polymorphism leading to a major change in the peptide mass thus inhibiting peptide identification in database search which depends on mass tolerance. In the 1683.77 Da peptide, it was not possible to determine the sequence up to N-terminus. However, the partial sequence determined was sufficient to show homology with TLP from tomato. A similar occurrence was found in all other de novo sequenced peptides.

The spots 1 and 2 have been identified as Actin and are isoforms of each other existing at a molecular weight of 45 kDa. Actin has been reported as an allergen in *Aspergillus fumigatus* [29], a shellfish named Clam [30] and shrimp [31]. It is one of the two major components involved in the muscle contraction. Actin also participates in many important cellular processes such as cellular motility, cytoplasmic streaming, and cellular signaling and devotes to the process of cell division. This is a highly conserved protein and could be easily identified through MASCOT search suggesting negligible amino acid substitutions in Actin from LC.

Spot 4, 5, 6 were identified as mitochondrial ATP synthase beta subunit and it is also evident that they are isoforms of each other as they possess similar molecular weight but different pIs. It is responsible for ATP synthesis and also participates as a novel plant cell death regulator protein. It was reported as an allergen from *Cannabis sativa* [32], *Ligustrum lucidum* [33] pollen grains and cow dander [34].

Spot 3, 7 and 8 demonstrated similarity with Thaumatin-like protein (TLP) from different plant species and could be isoforms of each other. These spots are part of the major allergenic region observed in 1D blot with individual sera as described previously. Since no other protein was found as an allergen in this region TLP can be recognized as a major allergen in LC pollen. TLPs are products of a large, highly complex gene family involved in plant defense response. TLP are also panallergens and has been found to be responsible for cross-reactivity amongst food and pollen grains [35]. As food allergen it has been reported in Apple [36], Peach [37], Olive [38], Kiwifruit [39], and Sapodilla [40] to name a few. Japanese Cedar [41], *Cupressus arizonica* [42], mountain cedar [43] pollen grains also harbor TLP allergens causing severe pollinosis in a Japanese cohort. These were found between a narrow MW range of 26–29 kDa whereas the pI varied between 4.2 and 6.5. In general, TLPs exist in between 20 and 30 kDa and have very compact 3D structure stabilized by 8 disulfide bridges. Peach TLP allergen was found to exist in three isoforms having pI ranging from 4.8 to 8.3. This implies that TLP undergoes considerable post-translational modifications causing such difference in isoelectric points, however, retaining its allergenic properties. TLP being a major allergen may show promise for being harnessed in component resolved diagnosis of LC pollen allergy.

Peptides from spot 9 showed significant homology to Glutamate decarboxylase. It catalyzes the conversion of glutamate to Gama Amino Butyric acid during the abiotic stress of plants and is identified as an allergen probably for the first time.

It was observed in some cases that peptides from each spot matched to a single type of protein though they are from different plant species. Since our identifications are based on homology, assignments to similar proteins across taxonomic restrictions are evident. Matching of a peptide to a protein suggests more homology in that region of the corresponding protein. In this study the presence of IgE reactivity on proteins are solely on the basis of linear epitopes as they are analyzed under denaturing conditions. Structural studies on individual allergens may shed light on the presence of conformational epitopes. Additionally, the allergens identified are only on the basis of IgE affinity. Experiments such as lymphoproliferation assays, purification of each of the allergens are required to describe their individual potencies in causing atopicity [44]. The peptides derived either from de novo sequencing or from database search can be used to design degenerate primers for the amplifying full-length gene of the allergens using Rapid Amplification of cDNA Ends (RACE) technique.

## Conclusions

Our study is probably the first comprehensive report on the identification of allergens from *Lantana camara* pollen which has a significant impact on the human health living within its vicinity. The combination of de novo sequencing and MS/MS based database search has led to an increased query coverage and can be used to identify allergens from other species having unknown genomes. Identification of the probable allergens in this study paves the way for developing recombinant hypoallergenic candidate vaccines, understanding allergen structure and its interaction with the immune system leading to better therapeutic interventions against Lantana pollen allergy.

### Ethics statement

The present study protocol was approved by the human ethics committee of Bose Institute and Indian primary respiratory care and allergy foundation, Kolkata. Informed written consents were obtained from patients and non-allergic volunteers for participation in the study. In case of minors, informed written consents were obtained from their guardians.

## Additional files

10.1186/s13223-016-0135-z Correlations of the most dominating species with the data from hospital and health survey. Correlations have been followed by linear regression analysis of those significant species which have most significant impact on human health of the area.
10.1186/s13223-016-0135-z Snapshots of the MASCOT search for all the peptides. Mascot scores of each peptide is given displaying their homology sequence coverage with other proteins of the other plant species.

## Abbreviations

1D: 1dimensional
2D: 2dimensional
ABC: ammonium bicarbonate
ATP: adenosine triphosphate
BLAST: basic local alignment search tool
DTT: dithiothreitol
EDTA: ethylenediaminetetraacetic acid
ELISA: enzyme-linked immunosorbent assay
IEF: isoelectric focusing buffer
kDa: kiloDalton
LC: *Lantana camara*
MALDI-TOF/TOF: matrix-assisted laser desorption/ionization—time of flight
MW: molecular weight
NBT/BCIP: nitro blue tetrazolium chloride/5-bromo-4-chloro-3-indolyl-phosphate
NCBInr: National Center for Biotechnology Information–non-redundant
pI: isoelectric point
PAM: percent accepted mutation
SDS-PAGE: sodium dodecyl sulfate polyacrylamide gel electrophoresis
sIgE: specific IgE
SIT: specific immunotherapy
TBST: tris-buffered saline tween-20
TLP: thaumatin-like protein
